The article "Effect of Different Repair and Reconstruction Methods Combined with Psychological Intervention on Quality of Life and Negative Emotion in Patients with Oral Cancer" was published in 2022. Journal: Comput Math Methods Med.

# Effect of Different Repair and Reconstruction Methods Combined with Psychological Intervention on Quality of Life and Negative Emotion in Patients with Oral Cancer

**DOI:** 10.1155/2022/7359584

**Published:** 2022-05-06

**Authors:** LinHu Wang, QingShan Dong, Mingfu Ye, Jiao Du, RongHua Zhou, XianHua Cai

**Affiliations:** ^1^Department of Stomatology, General Hospital of Central Theater Command of PLA, Wuhan 430070, China; ^2^Department of Orthopaedics, General Hospital of Central Theater Command of PLA, Wuhan 430070, China; ^3^Department of Oral Implantology, Stomatological Hospital of Xiamen Medical College, Xiamen Key Laboratory of Stomatological Disease Diagnosis and Treatment, Xiamen, 310068 Fujian, China; ^4^Oral and Maxillofacial Surgery, Wuhan Savaid Stomatology Hospital, Wuhan 430021, China

## Abstract

**Objective:**

To explore the effects of different repair and reconstruction methods combined with psychological intervention on the quality of life and negative emotion of patients with oral cancer.

**Methods:**

180 patients with oral cancer treated in our hospital from January 2018 to January 2020 were randomly divided into group A, group B, and group C, with 60 cases in each group. Group A and group B were repaired with submental island flap and free flap, respectively. Group C was divided into two groups, and group C was treated with routine nursing intervention. Group A and group B received psychological intervention. Clinical symptom scores, complication rate (CR), quality of life (according to the University of Washington quality of life questionnaire, UW-QOL), and negative emotion scores were compared.

**Results:**

After intervention, the clinical symptom scores and negative emotion scores of groups A and B were lower than those of group C (*P* < 0.001), as well as the CR (*P* < 0.05), and the UW-QOL scores of groups A and B were higher than those of group C (*P* < 0.05), but no significant differences in these aspects were presented between group A and group B (*P* > 0.05). The main factors affecting quality of life were swallowing/chewing, language, and saliva in group A; swallowing/chewing, language, and taste in group B; and appearance, swallowing/chewing, emotion, and language in group C.

**Conclusion:**

Psychological intervention can improve the mental state of patients with oral cancer after operation, optimize the effect of operation, and improve the quality of life. As the effect of psychological intervention on patients undergoing different repair and reconstruction methods is similar, it should be given according to patients' actual condition in the clinic.

## 1. Introduction

In recent years, the incidence rate of oral cancer has steadily increased. More than 300 thousand of the world's patients have oral cancer annually. There are more and more patients with surgical treatment. Although radical resection of oral cancer is advantageous in many aspects, it will damage the maxillofacial tissue of patients and affect the normal function and appearance, and some patients will suffer from a huge blow, resulting in more obvious mania, depression, and other negative emotions and greatly reducing their quality of life [1–3]. Nowadays, with the continuous optimization of relevant medical technology, oral cancer patients generally carry out repair and reconstruction in radical resection to improve their maxillofacial function. The most common repair and reconstruction methods in clinic include submental island flap transfer repair and free flap transfer repair, which is selected according to the maxillofacial defects of patients [4–7]. Psychological intervention is an important way to help patients rebuild their life beliefs, but there are few academic studies on different repair and reconstruction methods combined with psychological intervention.

The article "Effect of Different Repair and Reconstruction Methods Combined with Psychological Intervention on Quality of Life and Negative Emotion in Patients with Oral Cancer" was published in 2022. Journal: Comput Math Methods Med.

Based on this, to explore the effect of different repair and reconstruction methods combined with psychological intervention on the quality of life and negative emotion of patients with oral cancer, 180 oral cancer patients admitted to our hospital from January 2018 to January 2020 were selected as the research object.

## 2. Materials and Methods

### 2.1. General Information

180 oral cancer patients admitted to our hospital from January 2018 to January 2020 were selected as the research object and equally divided into groups A, B, and C, with 60 cases in each group. There is no significant difference in patients' general information (*P* > 0.05); see Table 1.

### 2.2. Inclusion Criteria

The inclusion criteria of the study were as follows: ① patients or their family members fully understood the study process and signed the informed consent; ② patients were confirmed as having oral cancer by pathology; ③ patients had undergone repair and reconstruction after radical resection of oral cancer; and ④ this study as approved by the hospital ethics committee, and all patients signed the informed consent.

### 2.3. Exclusion Criteria

The exclusion criteria for patients of the study were as follows: ① presence of mental problems or inability to communicate with others, ② suffering from other organic diseases, ③ recurrence of the disease, and ④ prior chemoradiotherapy before operation.

### 2.4. Methods

Group A and group B were treated with submental island flap transplantation and free flap transplantation, respectively, group C was treated with half an operation, and group C was treated with routine nursing. Group A and group B received psychological intervention. The methods for operation and nursing intervention were as follows.

The article "Effect of Different Repair and Reconstruction Methods Combined with Psychological Intervention on Quality of Life and Negative Emotion in Patients with Oral Cancer" was published in 2022. Journal: Comput Math Methods Med.

#### 2.4.1. Submental Island Flap Transfer Repair

① The flap was designed according to patients' chin skin condition and wound condition, and the lower edge of the mandible and 10 mm from the lower edge of the hyoid bone were marked as the incisions of upper and lower margin of the flap. ② The platysma muscle was cut to separate the marginal mandibular branch of facial nerve and submental artery and vein pedicle of facial artery and vein according to the marking line of upper margin. ③ The prepared flap was transferred to the defect for repair after the vascular pedicle of the myocutaneous flap was fully free, and then, the tissue around submental skin was sutured.

#### 2.4.2. Free Flap Transfer Repair

① The flap was designed according to the forearm skin condition and repair condition of patients, and the middle points of forearm cephalic vein and radial artery were connected to form the middle line of flap transfer. ② When performing the radical resection of oral cancer, the radial forearm flap was taken out, and the skin was cut from the distal end to free the cephalic vein and radial vascular pedicle. ③ The prepared flap was transferred to the defect for repair, the vascular end anastomosis was leveled, and then, the donor site was covered with middle-thick skin of abdomen for suture.

#### 2.4.3. Nursing Intervention

Routine nursing: nursing staff paid attention to patients' sign data and help patients with their oral care to maintain fine flap condition and avoid wound infection.

Psychological intervention: ① psychological health education and training were given to nursing staff to ensure scientific and highly effective communication with patients and solving patients' psychological problems; evidence-based conferences were also held to conclude the common psychological problems and work out basic solution by analyzing the real living condition of patients with oral cancer so that psychological intervention was based on evidence. ② Nursing staff informed patients about the cause of oral cancer and gave patients a full understanding of their conditions and, at the same time, explained the differences and precautions of various treatments according to patients' actual condition and the repair and reconstruction method selected to enhance the self-control ability. ③ Nursing staff were familiar with patients' information and conducted living guidance to patients with history of drinking and smoking so that such patients understood that alcohol and cigarette were the key factors affecting the reconstruction effect; meanwhile, nursing staff also increased patients' intake of high-protein foods to provide nutrition for recovery. ④ Nursing staff increased the frequency of communicating with patients' family members on basic oral nursing methods so that effective home nursing was provided scientifically and effectively, patients' daily life was monitored, and patients' oral condition was improved comprehensively. ⑤ Nursing staff increased the frequency of communicating with patients by putting themselves into patients' condition with narrative medicine and being considerate to solve problems for patients; and prompt intervention was warranted in patients presenting with significant psychiatric symptoms.

The article "Effect of Different Repair and Reconstruction Methods Combined with Psychological Intervention on Quality of Life and Negative Emotion in Patients with Oral Cancer" was published in 2022. Journal: Comput Math Methods Med.

### 2.5. Observation Criteria

① Comparison of clinical symptom scores: symptoms included insomnia, nausea and vomiting, pain, fatigue, and diarrhea and were rated (on a 0-100 scale) by reference to the visual analogue scale (VSA) for pain, with lower scores indicating less symptoms

② Comparison of CR: complications included incision infection, necrosis of skin flap, wound bleeding, and stress ulcer

③ Comparison of UW-QOL scores: the score was rated based on the University of Washington Quality of Life Questionnaire (UW-QOL) of head and neck cancer patients on a scale of 0-100, with lower scores indicating worse quality of life [8–11]

④ Investigation on factors affecting patients' quality of life, which was carried out by self-designed questionnaire

⑤ Comparison of negative emotion scores of patients after intervention. The scores (on a scale of 0-100) of patients' self-rating anxiety scale (SAS) and self-rating depression scale (SDS) were compared, with higher scores indicating heavier negative emotion [12–15]

### 2.6. Statistical Processing

In this study, the data processing software was SPSS 20.0, the picture drawing software was GraphPad Prism 7 (GraphPad Software, San Diego, USA), items included were enumeration data and measurement data, methods used were the *χ*^2^ test and *t*-test, and differences were considered statistically significant at *P* < 0.05.

## 3. Results

### 3.1. Comparison of Patients' Clinical Symptom Scores

The clinical symptom scores of group A and group B were significantly lower than those of group C (*P* < 0.001), but no significant difference was presented between group A and group B (*P* > 0.05); see Table 2.

### 3.2. Comparison of Patients' CR

The CR of group A and group B was significantly lower than that of group C (*P* < 0.05), but no significant difference was presented between group A and group B (*P* > 0.05), see Figure 1.

Note: in Figure 1, the black area showed incision infection, the dark gray area showed necrosis of skin flap, the light gray area showed wound bleeding, the yellow area showed stress ulcer, and the green area showed no complications; and from left to right, they were group A, group B, and group C.

The article "Effect of Different Repair and Reconstruction Methods Combined with Psychological Intervention on Quality of Life and Negative Emotion in Patients with Oral Cancer" was published in 2022. Journal: Comput Math Methods Med.

The number of patients with incision infection in groups A, B, and C was 1, 1, and 3, respectively.

The number of patients with necrosis of skin flap in groups A, B, and C was 1, 2, and 4, respectively.

The number of patients with wound bleeding in groups A, B, and C was 1, 0, and 3, respectively.

The number of patients with stress ulcer in groups A, B, and C was 0, 1, and 2, respectively.

The number of patients with no complications in groups A, B, and C was 57, 56, and 48, respectively.

### 3.3. Comparison of Patients' UW-QOL Scores

After intervention, the UW-QOL scores of group A and group B were significantly higher than those of group C (*P* < 0.05), but no significant difference was presented between group A and group B (*P* > 0.05); see Table 3.

### 3.4. Investigation on Factors Affecting Patients' Quality of Life

The main factors affecting quality of life were swallowing/chewing, language, and saliva in group A; swallowing/chewing, language, and taste in group B; and appearance, swallowing/chewing, emotion, and language in group C; see Table 4.

### 3.5. Comparison of Patients' Negative Emotion Scores after Intervention

After intervention, the negative emotion scores of group A and group B were significantly lower than those of group C (*P* < 0.001), but no significant difference was presented between group A and group B (*P* > 0.05); see Figures 2 and 3.

## 4. Discussion

Patients with oral cancer usually have maxillofacial tissue injury after radical resection. Immediate suture after operation will lead to physical and mental disorders and great survival pressure. At present, it is advocated in the academic community that repair and reconstruction should be applied directly after radical resection of oral cancer, so as to repair the maxillofacial defects of patients, and then comprehensively optimize the surgical effect and reduce the life difficulty of patients [16–19]. After the repair and reconstruction, the maxillofacial region of patients cannot be restored to its original state, and some patients still have serious depression tendency and even extreme behaviors such as suicide in case of complications including incision infection. Therefore, it is necessary to intervene in psychological intervention measures to reduce the possibility of medical malignant events through scientific and efficient nursing means [20–23].

In this study, the clinical symptom scores and negative emotion scores of group A and group B after intervention were lower than those of group C, as well as the CR, of which the reason was that nursing staff enhanced patients' and their family members' understanding of oral cancer to improve the self-protection ability of patients and lower the possibility of complications with quality nursing at home. In addition, nursing staff learned professional psychological knowledge from special psychological education and training, which fully promoted the psychological intervention in a more scientific and effective way, so as to practically solve patients' mental problems during communication. Therefore, patients in group A and group B had better mental condition and recovered faster.

The article "Effect of Different Repair and Reconstruction Methods Combined with Psychological Intervention on Quality of Life and Negative Emotion in Patients with Oral Cancer" was published in 2022. Journal: Comput Math Methods Med.

After intervention, the UW-QOL scores of group A and group B were higher than those of group C, and with analysis, the main factors affecting the quality of life were swallowing/chewing, language, and saliva in group A; swallowing/chewing, language, and taste in group B; and appearance, swallowing/chewing, emotion, and language in group C. Compared with the other two groups, emotion and appearance were additional factors in group C, which was due to the fact that patients in group C lacked effective psychological counseling, suffered from heavier metal stress, and had their daily life affected adversely by mental factors [24]. In the scholar Davudov et al.'s study, oral cancer patients undergoing repair and reconstruction were divided into groups according to whether they were given psychological nursing or not, and it was concluded that patients in the nursing group achieved the UW-QOL score of 83.55 ± 6.56, which was significantly higher than the control group [25], indicating that psychological nursing was an important way to improve patients' quality of life.

It is worth noting that in this study, no significant difference was showed between group A and group B, but the indicators of group A were slightly better than those of group B due to the possible reason that patients with submental island flap transfer repair usually had slighter maxillofacial damage, less physical and mental pressure, and better basic condition.

In conclusion, different repair and reconstruction methods combined with psychological intervention can effectively improve the negative emotion and the quality of life for oral cancer patients, which should be promoted and applied in clinical practice. As the effect of psychological intervention on patients undergoing different repair and reconstruction methods is similar, it should be given according to patients' actual condition in the clinic.

## Figures and Tables

**Figure 1:** Comparison of patients' CR.

The article "Effect of Different Repair and Reconstruction Methods Combined with Psychological Intervention on Quality of Life and Negative Emotion in Patients with Oral Cancer" was published in 2022. Journal: Comput Math Methods Med.

**Figure 2:** Comparison of patients' SAS scores (^−^*x* ± *s*, points). Note: the horizontal axis from left to right showed group A, group B, and group C, and the vertical axis showed the SAS score (points). The SAS score of group A, group B, and group C was 28.12 ± 2.56, 28.89 ± 2.11, and 35.89 ± 5.65, respectively. ∗ indicated *P* < 0.001 when comparing among the groups.

**Figure 3:** Comparison of patients' SDS scores (^−^*x* ± s, points). Note: the horizontal axis from left to right showed group A, group B, and group C, and the vertical axis showed the SDS score (points). The SDS score of group A, group B, and group C was 32.56 ± 3.44, 32.78 ± 3.56, and 40.02 ± 3.87, respectively. ∗ indicated *P* < 0.001 when comparing among the groups.

**Table 1:** Comparison of patients' general information.

Group	Sex ratio	Age (years old)	BMI (kg/m^2^)	History of drinking and smoking		Complication	
				Yes	No	Yes	No
Group A	45/15	54.89 ± 8.26	24.12 ± 2.21	28	32	12	48
Group B	46/14	55.01 ± 8.24	24.14 ± 2.23	28	32	13	47
Group C	44/16	54.99 ± 8.32	24.10 ± 2.25	27	33	11	49

**Table 2:** Comparison of patients' clinical symptom scores (^−^*x* ± *s*, points).

Group	Group A	Group B	Group C
Insomnia	50.21 ± 5.23^∗^	51.56 ± 5.87^∗^	61.23 ± 6.45
Nausea and vomiting	52.56 ± 4.51^∗^	53.12 ± 5.46^∗^	62.45 ± 6.12
Pain	49.32 ± 3.56^∗^	50.45 ± 6.52^∗^	59.23 ± 6.50
Fatigue	49.11 ± 4.52^∗^	50.12 ± 6.23^∗^	59.89 ± 5.78
Diarrhea	51.22 ± 3.56^∗^	52.00 ± 3.47^∗^	60.11 ± 4.58

∗ indicated *P* < 0.001 when comparing with group C.

**Table 3:** Comparison of patients' UW-QOL scores (^−^*x* ± *s*, points).

Time	Group A	Group B	Group C
Before intervention	43.56 ± 5.56	43.10 ± 5.78	42.78 ± 5.45
After intervention	82.45 ± 6.23^∗^	81.11 ± 5.78^∗^	55.56 ± 4.89
*t*	36.076	36.019	13.520
*P*	<0.001	<0.001	<0.001

∗ indicated *P* < 0.001 when comparing with group C.

**Table 4:** Investigation on factors affecting patients' quality of life.

Item	Group A		Group B		Group C	
	*N*	Proportion (%)	*N*	Proportion (%)	*N*	Proportion (%)
Pain	5	8.3	6	10.0	5	8.3
Appearance	0	0.0	1	1.7	10	16.7
Vigor	1	1.7	2	3.3	1	1.7
Entertainment	2	3.3	1	1.7	5	8.3
Swallowing/chewing	18	30.0	18	30.0	12	20.0
Language	18	30.0	16	26.7	7	11.7
Shoulder function	2	3.3	2	3.3	1	1.7
Taste	2	3.3	10	16.7	4	6.7
Saliva	12	20.0	4	6.7	5	8.3
Emotion	0	0.0	0	0.0	10	16.7

## Data Availability

The datasets during the current study are available from the corresponding author on reasonable request.
